RETRACTED

# Effect of Targeted Care plus Exercise Intervention on Blood Glucose Levels and Maternal and Newborn Outcomes in Patients with Gestational Diabetes Mellitus

**DOI:** 10.1155/2022/7584936

**Published:** 2022-09-27

**Authors:** Xiufang He, Xiaqing Geng, Manting Sha, Yan Jia, Gaiying Cui

**Affiliations:** ^1^First Department of Obstetrics, Shijiazhuang Obstetrics and Gynecology Hospital, Shijiazhuang, Hebei, China; ^2^Nursing Department, Shijiazhuang Fourth Hospital, Shijiazhuang, Hebei, China; ^3^Seventh Department of Obstetrics, Shijiazhuang Fourth Hospital, Shijiazhuang, Hebei, China; ^4^Third Department of Obstetrics, Shijiazhuang Fourth Hospital, Shijiazhuang, Hebei, China; ^5^Ward Management Center, Shijiazhuang Fourth Hospital, Shijiazhuang, Hebei, China

## Abstract

**Objective:**

To evaluate the effect of targeted care plus exercise intervention on blood glucose levels and maternal and newborn outcomes in patients with gestational diabetes mellitus (GDM).

**Methods:**

A total of 96 patients with GDM admitted to our hospital between March 2018 and January 2020 were recruited and assigned to receive either routine nursing (routine group) or targeted care plus exercise intervention (study group) via random method, with 48 patients in each group. Outcome measures included blood glucose, immune function, maternal and newborn outcome, and nursing satisfaction.

**Results:**

The patients in the study group had significantly lower amniotic fluid index (AFI), weight at delivery, body mass index (BMI), and weight gain during pregnancy than patients in the routine group (*P* < 0.05). There was no statistically significant difference in blood glucose between the two groups of patients before the intervention (*P* > 0.05). Targeted care plus exercise intervention resulted in significantly lower levels of fasting blood glucose (FBG), 2 h postprandial blood glucose (2hPBG), and blood glucose before bed versus routine care (*P* < 0.05). The patients with targeted care plus exercise intervention had higher immunoglobulin G (IgG) and IgM levels; higher CD3+, CD4+, and CD8+ levels; and lower lgA levels versus those with routine care (*P* < 0.05). Targeted care plus exercise intervention was associated with a lower incidence of negative pregnancy outcomes and a higher satisfaction versus routine care (*P* < 0.05).

**Conclusion:**

Targeted treatment plus exercise intervention efficiently controls blood glucose levels in GDM patients, improves immunological function, lowers the risk of pregnancy problems, improves pregnancy outcomes, and promotes patient satisfaction, indicating a high potential for therapeutic development. Targeted treatment combined with exercise intervention is encouraged following effective pharmacological interventions to facilitate recovery.

RETRACTED

## 1. Introduction

Diabetes mellitus is a metabolic disease characterized by hyperglycemia. Hyperglycemia is caused by insufficient insulin secretion and/or impaired biological activity and causes chronic damage and dysfunction of the kidneys, heart, blood vessels, and nerves. During pregnancy, maternal metabolism, system function, and skeletal changes are noticed. Gestational diabetes mellitus (GDM) [1] is frequent pregnancy comorbidity that refers to diabetes mellitus that develops solely during pregnancy, with normal glucose metabolism or potentially decreased glucose tolerance prior to pregnancy. According to relevant epidemiological statistics, the incidence of GDM is 1%-14% globally and 1%-5% in China in the past two decades, with a significant increasing trend [2]. The pathogenesis is usually because the nutritional requirements of the fetus increase with gestational age and that glucose obtained from the mother through the placenta is the main source of energy for the fetus.

Renal plasma flow and glomerular filtration increase during pregnancy, with less elastic renal tubular reabsorption of glucose, thereby causing increased stress on glucose metabolism in vivo [3, 4]. Maternal placental prolactin, estrogen, progesterone, cortisol, and placental insulinase rise in the second trimesters, but insulin sensitivity declines with increasing gestational age, and blood glucose fails to adapt to this physiological change, leading to GDM [5]. Previous studies have confirmed an association of GDM with poor pregnancy outcomes, which poses a great threat to the health of the pregnant woman and the newborn. The common clinical treatment of gestational diabetes includes pharmacological control, dietary and nutritional control, and exercise interventions [6, 7]. Lifestyle interventions are essential in the comprehensive management of diabetes. Exercise can effectively increase the body's sensitivity to insulin and maintain blood glucose stability, and its positive role in preventing the onset and development of diabetes is receiving increasing attention [8].

In addition, the physiological and psychological changes of pregnant women during hospitalization can affect their compliance behavior and confidence in fetal preservation. Conventional care does not pay attention to the emotional factors of the patients and the role of their family members. In recent years, it has been found that women during pregnancy are most dependent on family members for life and psychological support, which yields a strong positive impact on the pregnant woman. It has been reported that improvement in the care of GDM patients contributes to enhancing treatment outcomes and pregnancy outcomes [9]. Targeted care provides effective clinical treatment and has significant advantages in postillness care. Accordingly, this study was to evaluate the effect of targeted care plus exercise intervention on blood glucose levels and maternal and newborn outcomes in patients with GDM, so as to provide clinical references.

RETRACTED

## 2. Materials and Methods

### 2.1. Participants

A total of 96 patients with GDM admitted to our hospital between March 2018 and January 2020 were recruited and assigned to receive either routine nursing (routine group) or targeted care plus exercise intervention (study group), with 48 patients in each group. All included patients were female, aged 26-36 (28.97 ± 3.62) years.

#### 2.1.1. Random Method

The randomization was carried out using an online web-based randomization tool (freely available at http://www.randomizer.org/). For concealment of allocation, the randomization procedure and assignment were managed by an independent research assistant who was not involved in the screening or evaluation of the participants.

#### 2.1.2. Sample Size Estimation

For sample size calculation, the sample size was determined according to the hospital sampling survey case-control study method, the estimated prevalence was 5%; the relative error of the sampling survey was 20% and set at 1.5, with a 95% confidence interval, Za = 1.96, and a 10% data incompleteness rate; and the final calculated sample size was in the range of 35 to 50.

#### 2.1.3. Ethical Considerations

The trial was conducted according to Good Clinical Practice guidelines developed by the International Council for Harmonisation and in compliance with the trial protocol. The protocol was approved by the institutional review boards of Shijiazhuang Fourth Hospital (Ethics No. E297391). All patients provided written informed consent per the Declaration of Helsinki principles. An independent data monitoring committee monitored safety and efficacy data.

### 2.2. Inclusion and Exclusion Criteria

#### 2.2.1. Inclusion Criteria

Patients who met the relevant diagnostic criteria for gestational diabetes in the IADPSG 2010 and were diagnosed with gestational diabetes [10], with singleton pregnancies, and who provided written informed consent were included.

#### 2.2.2. Exclusion Criteria

Patients with other gynecological diseases, with hypertension and heart disease, with unconsciousness that prevented normal communication, with malignant tumors and circulatory system diseases, with hospital referrals, or who revoked their consent were excluded.

### 2.3. Treatment Methods

Patients in the routine group received routine care, including health education, life care, nutritional guidance, medication guidance, and prevention of complications, such as regular checks of maternal and fetal status, low-glycemic diet instruction, insulin therapy, and monitoring of drug reactions.

RETRACTED

Patients in the study group were given targeted care plus exercise intervention. (1) Establishment of a health education team: a health education team consisting of obstetricians and gynecologists, endocrinologists, nutritionists, and psychologists was established to promote disease knowledge and raise the patient's disease and treatment awareness through multimedia methods. (2) Psychological care: to minimize negative emotions, the nursing team maintained active communication with patients and encouraged them to share their sentiments so as to strengthen patients' trust in the nursing staff, thereby improving patient compliance with nursing management. (3) Exercise intervention: the patient's physical condition and dietary habits were identified, and an individual exercise program tailored to the patient was developed, with appropriate daily training duration and intensity. In addition, the nursing staff communicated and coordinated with the patients and their families on admission to explain the benefits of physical exercise in improving the physical function of GDM patients. (4) Infection prevention: infection prevention included daily monitoring of body temperature, timely change of clothes and bedding, cleaning the perineum with acidic soap, wearing loose clothing, strict prohibition of sexual intercourse for 42 days, at least 30 minutes of daily ultraviolet radiation, and maintenance of indoor ventilation.

All patients received dietary instructions [11], including the development of personalized, diverse, and scientific nutritional dietary recipes, increased intake of high-quality protein and dietary fiber, regular monitoring of blood glucose and body weight, and timely adjustment of dietary regimens.

### 2.4. Outcome Measures

1. Clinical indices: the relevant clinical indices, including amniotic fluid index (AFI), weight at delivery, body mass index (BMI), and weight gain during pregnancy, were recorded
2. Blood glucose level: venous blood was collected from the patients before and after the intervention to determine the fasting blood glucose (FBG), 2 h postprandial blood glucose (2hPBG), and blood glucose before bed by an AU5800 automatic biochemical analyzer
3. Immunological function: the levels of immunoglobulin G (IgG), immunoglobulin A (lgA), and immunoglobulin M (IgM) in the peripheral blood of the two groups of neonates were determined by ELISA. The levels of T-cell subsets CD3+, CD4+, and CD8+ were measured by Partee flow cytometry in the two groups of neonates. Higher levels of T-cell subsets indicate better intervention outcomes
4. Pregnancy outcomes: the mode of delivery and outcomes of pregnancy in both groups was recorded in detail, including preterm delivery, cesarean delivery, macrosomia, excessive amniotic fluid, and premature rupture of membranes, and the incidence of negative pregnancy outcomes was calculated for comparison between groups
5. Nursing satisfaction: the nursing satisfaction questionnaire (including the attitude of medical staff, efficiency of medical staff, and health education quality by medical staff) created by our hospital was divided into four levels (highly satisfied, satisfied, less satisfied, and dissatisfied) to understand the satisfaction of patients in both groups

RETRACTED

### 2.5. Statistical Analysis

If the parameter beta is either a difference of means, a log odds ratio, or a log hazard ratio, then it is reasonable to assume that *b* is unbiased and normally distributed. The GraphPad Prism 8 software was used to plot the graphics, and the SPSS 22.0 software was used for data analyses. The count data were expressed as (*n* (%)) and analyzed using the chi-square test. The measurement data were expressed as mean ± standard deviation and analyzed using the *t*-test. *P* < 0.05 was considered the cut-off for statistical significance.

## 3. Results

### 3.1. Patient Characteristics

In the routine group, there were 48 patients, aged 26-35 (28.86 ± 3.68) years, with a gestational week of 32-39 (36.35 ± 2.36) weeks and parity of 0-3 (1.01 ± 0.32). In the study group, there were 48 patients, aged 28-36 (29.03 ± 3.14) years, with a gestational week of 32-38 (36.18 ± 2.17) weeks and parity of 0-3 (1.08 ± 0.34). The patient characteristics between the two groups were comparable (*P* > 0.05) (Table 1).

### 3.2. Clinical Indices

The patients in the study group had significantly lower AFI, weight at delivery, BMI, and weight gain during pregnancy than patients in the routine group (*P* < 0.05) (Table 2).

### 3.3. Blood Glucose

There was no statistically significant difference in blood glucose between the two groups of patients before the intervention (*P* > 0.05). After the intervention, the blood glucose levels of patients in both groups decreased, with lower levels of FBG, 2hPBG, and blood glucose before bed in the study group than in those in the routine group (*P* < 0.05) (Table 3).

### 3.4. Immune Function

The patients in the study group had higher IgG and IgM levels (10.25 ± 1.32 and 0.38 ± 0.13) than those in the conventional group (6.52 ± 1.12 and 0.25 ± 0.06) and lower lgA levels (0.41 ± 0.11) than those in the routine group (0.53 ± 0.22). The levels of CD3+, CD4+, and CD8+ were higher in the study group than in the routine group (*P* < 0.05) (Table 4).

RETRACTED

### 3.5. Pregnancy Outcome

In the study group, there were 2 (4.67%) cases of preterm delivery, 5 (10.42%) cases of cesarean delivery, 1 (2.08%) case of macrosomia, 2 (4.67%) cases of excess amniotic fluid, and 1 (2.08%) case of premature rupture of membranes. In the routine group, there were 10 (20.83%) cases of preterm delivery, 24 (50.00%) cases of cesarean delivery, 7 (14.58%) cases of macrosomia, 9 (18.75%) cases of excess amniotic fluid, and 7 (14.58%) cases of premature rupture of membranes. Targeted care plus exercise intervention was associated with a lower incidence of negative pregnancy outcomes versus routine nursing (*P* < 0.05) (Table 5).

### 3.6. Nursing Satisfaction

In the routine group, 11 (24.44%) patients were highly satisfied, 25 (52.08%) were satisfied, 9 (18.75%) were less satisfied, and 4 (8.33%) were dissatisfied. In the study group, 20 (41.67%) patients were highly satisfied, 25 (52.08%) were satisfied, 2 (4.17%) were less satisfied, and 1 (2.08%) was dissatisfied. The total satisfaction of patients in the study group (93.75%) was significantly higher than that of the conventional group (72.92%) (*P* < 0.05) (Figure 1).

## 4. Discussion

Diabetes presents a slow progression with high complications and serious conditions that are life-threatening to the patient. GDM patients are predisposed to significant vasculopathy, thickening of the vascular endothelium, narrowing of the lumen, and inadequate blood flow to the tissues, resulting in hypertensive problems during pregnancy, fetal growth limitation, and maternal renal failure. Furthermore, the fetus with GDM is exposed to a hyperglycemic situation that predisposes to greater risks of macrosomia and cesarean birth, and 20%-50% of GDM patients have poor medication adherence. Nursing interventions [12] are mostly used in the management of diabetic patients to strictly manage their blood glucose and provide assistance in lifestyle adjustment, proper diet control, and appropriate exercise [13].

It has been indicated that appropriate exercise could improve the sensitivity of body tissues to insulin and increase the utilization of glucose by muscle tissues [14]. Rehabilitation care refers to a series of targeted rehabilitation training programs developed by medical and nursing staff according to the results of disease assessment after the patient reaches the stable stage of the disease to achieve rapid recovery. Exercise training interventions rapidly improve the exercise endurance of patients and enhance their physical fitness, thus facilitating the smooth implementation of treatment and care and improving clinical outcomes. Targeted care involves an organic combination of health education, diet, and exercise to provide effective infection prevention, reduce maternal complications, and improve pregnancy outcomes [15].

RETRACTED

In the present study, 96 patients with GDM were recruited to investigate the effects of targeted care plus exercise intervention on blood glucose levels and pregnancy outcomes in patients with GDM.

The results showed that the AFI, weight at delivery, BMI, and weight gain during pregnancy in the study group were significantly lower than those in the routine group, and after the intervention, the blood glucose levels in both groups decreased, with lower levels of FBG, 2hPBG, and blood glucose before bed in the study group, suggesting a better performance of targeted care plus exercise intervention versus routine nursing. The rationale for this is that targeted care formulates individualized care schemes based on patients' real situations, and its combination with exercise treatments delivers refined and standardized management of patients' everyday lives [16], thereby providing effective blood glucose control. Previous studies suggest that GDM is associated with reduced cellular immune function in patients and that immunoglobulin and T-lymphocyte levels effectively reflect the immune status of the body. The results of the present study revealed that patients in the study group had higher levels of IgG, IgM, CD3+, CD4+, and CD8+ and lower levels of IgA than those in the routine group. Thyroxine, adrenaline, and hormones are actively secreted when bodily functions change throughout pregnancy, and the active hormonal changes impact blood glucose fluctuations, considerably increasing the risk of GDM in pregnancy. Clinical evidence suggests that GDM raises the risk of infection in pregnant women and fetuses and that dietary restriction is essential for disease management. Here, all patients were given dietary guidance [17], and patients in the study group received targeted care plus exercise intervention, including more detailed and thorough nutritional dietary recipes; regular monitoring of weight, lipid, and blood glucose changes and nutritional outcomes; appropriate adjustment of patients' dietary plans; and individual exercise plans [18] to improve patients' physical fitness, thereby effectively enhancing their immune function. This is consistent with Miko's study findings, which demonstrated that scientific nutritional and dietary treatments, as well as reasonable and effective exercise, could successfully manage pregnant women's blood lipids and blood glucose levels, as well as greatly increase their immunity.

RETRACTED

It has been reported that GDM patients with poor glycemic control deliver newborns with poorer health than those with well-controlled glycemia. The results of the present study showed that the study group had a lower incidence of preterm delivery, cesarean delivery, macrosomia, excess amniotic fluid, and premature rupture of membranes than the control group, indicating that targeted nursing plus exercise interventions improved maternal and newborn outcomes. Obesity is one of the leading causes of hyperglycemia during pregnancy, which alters fetal blood glucose levels and causes delivery problems. Appropriate regular exercise in patients substantially improves glucose tolerance and insulin resistance in patients with gestational diabetes and markedly reduces glycemic control by reducing insulin requirements, thereby improving maternal and infant outcomes [19, 20]. Targeted care allows health care providers to communicate more with patients during the process of health education, which results in greater patient trust and improved cooperation with treatment. Through basic education, diet education, and blood glucose monitoring, patients have a deeper understanding of their condition, and their self-management awareness can be improved simultaneously [21, 22]. Moreover, patients in the study group were more satisfied with the nursing than those in the control group, which is attributed to the better pregnancy outcomes and timely management of negative emotions through the joint intervention of targeted nursing and exercise therapy [23].

This study provides an alternative treatment option for future patients with gestational diabetes through clinical observation. Targeted care plus exercise intervention modulates patients' blood glucose levels and maternal and infant outcomes. It provides insights for future clinical diagnosis and treatment, as well as directions for the design of future matching medications. There are also limitations in the present study. First, the study sample size was small, the follow-up time was short, and the length of observation was insufficient for such a complex mechanism of change as diabetes. Future studies will expand the sample size, extend the observation time, increase the observation index, control the influencing factors, and eliminate the drawbacks to produce more accurate research results. In current basic and clinical studies, more and more possible pathways and biomarkers affecting diabetic pregnancy have been confirmed, providing more potential targets for drug research and indicating the direction of exploration to improve the prognosis of diabetic pregnancy patients. It is expected that more drugs to improve patients' quality of life will be developed in the future based on such studies, offering more therapeutic possibilities for the clinical management of GDM.

RETRACTED

## 5. Conclusion

Targeted care plus exercise intervention effectively regulates blood glucose levels in patients with GDM, effectively enhances immune function, reduces the risk of pregnancy complications, improves pregnancy outcomes, and increases patient satisfaction, which demonstrates great potential for clinical promotion.

## Figures and Tables

**Figure 1:** Nursing satisfaction. The total satisfaction of patients in the study group (93.75%) was significantly higher than that of the conventional group (72.92%). Note: ∗ indicates a significant difference between the two groups in terms of nursing satisfaction.

**Table 1:** Patient characteristics ($\bar{x}\pm s$).

Group	*n*	Age		Gestational week		Parity	
		Range	Mean	Range	Mean	Range	Mean
Routine	48	26-35	28.86 ± 3.68	32-39	36.35 ± 2.36	0-3	1.01 ± 0.32
Study	48	28-36	29.03 ± 3.14	32-38	36.18 ± 2.17	0-3	1.08 ± 0.34
*t*	—	—	0.243	—	0.367	—	1.039
*P* value	—	—	0.809	—	0.714	—	0.301

**Table 2:** Clinical indices ($\bar{x}\pm s$).

Group	*n*	Amniotic fluid index	Weight at delivery (kg)	BMI (kg/m^2^)	Weight gain during pregnancy (kg)
Routine	48	124.35 ± 16.85	71.01 ± 2.15	21.26 ± 0.78	17.99 ± 5.92
Study	48	105.87 ± 15.33	66.98 ± 2.85	20.17 ± 0.52	16.01 ± 3.51
*t*	—	5.620	7.821	8.056	1.992
*P* value	—	<0.001	<0.001	<0.001	0.049

**Table 3:** Blood glucose ($\bar{x}\pm s$).

	Indices	Routine (*n* = 48)	Study (*n* = 48)	*t*	*P* value
Before intervention	FBG	7.01 ± 1.68	7.04 ± 1.53	0.091	0.928
	2hPBG	10.12 ± 2.08	10.11 ± 2.09	0.023	0.982
	Blood glucose before bed	7.56 ± 1.37	7.63 ± 1.21	0.265	0.792
After intervention	FBG	5.87 ± 0.69^∗^	5.05 ± 0.58^∗^	6.303	<0.001
	2hPBG	7.62 ± 0.76^∗^	6.91 ± 0.62^∗^	5.015	<0.001
	Blood glucose before bed	6.68 ± 0.74^∗^	6.08 ± 0.71^∗^	4053	<0.001

Note: ∗ indicates a significant difference between the pre- and posttreatment in the same group. FBG: fasting blood glucose; 2hPBG: 2 h postprandial blood glucose.

**Table 4:** Immune function ($\bar{x}\pm s$).

	Indices	Routine (*n* = 48)	Study (*n* = 48)	*t*	*P* value
Immunoglobulin (g/L)	IgG	6.52 ± 1.12	10.25 ± 1.32	14.928	<0.001
	lgA	0.53 ± 0.22	0.41 ± 0.11	3.308	0.001
	IgM	0.25 ± 0.06	0.38 ± 0.13	6.291	<0.001
T lymphocytes (%)	CD3^+^	45.84 ± 8.61	53.41 ± 9.47	4.098	<0.001
	CD4^+^	23.48 ± 4.15	38.48 ± 7.14	12.584	<0.001
	CD8^+^	14.15 ± 4.26	26.17 ± 7.23	9.924	<0.001

**Table 5:** Pregnancy outcomes (%).

Group	*n*	Preterm delivery	Cesarean delivery	Macrosomia	Excess amniotic fluid	Premature rupture of membranes
Routine	48	10 (20.83)	24 (50.00)	7 (14.58)	9 (18.75)	7 (14.58)
Study	48	2 (4.67)	5 (10.42)	1 (2.08)	2 (4.67)	1 (2.08)
*x* ^2^	—	6.095	17.836	4.909	5.031	4.909
*P* value	—	0.014	<0.001	0.027	0.025	0.027

RETRACTED

## Data Availability

All data generated or analyzed during this study are included in this published article.
